# Overexpression of Suprabasin is Associated with Proliferation and Tumorigenicity of Esophageal Squamous Cell Carcinoma

**DOI:** 10.1038/srep21549

**Published:** 2016-02-22

**Authors:** Jinrong Zhu, Geyan Wu, Qingyuan Li, Hui Gong, Junwei Song, Lixue Cao, Shu Wu, Libing Song, Lili Jiang

**Affiliations:** 1 Department of Pathophysiology, Guangzhou Medical University, Guangzhou, Guangdong 511436 China; 2 Department of Experimental Research, State Key Laboratory of Oncology in Southern China, Sun Yat-sen University Cancer Centre, Guangzhou, 510060, China; 3 Department of Biochemistry, Zhongshan School of Medicine, Sun Yat-sen University, Guangzhou, Guangdong 510080, China; 4 Guangdong Country Garden School, Shunde, Foshan, Guangdong 528312, China; 5 Central Laboratory, Nanshan Hospital, Guangdong Medical University, Shenzhen, Guangdong, 518052, China

## Abstract

Suprabasin is a recently identified oncoprotein that is upregulated in multiple cancers. However, the clinical significance and biological role of suprabasin in human esophageal squamous cell carcinoma (ESCC) remains unclear. In the current study, we reported that suprabasin was markedly overexpressed in ESCC cell lines and tissues at both mRNA and protein levels, and this was associated with advanced clinical stage, tumor-nodes-metastasis (TNM) classification, histological differentiation, tumor size and poorer survival. Furthermore, we found that both proliferation and tumorigenicity of ESCC cells were significantly induced by suprabasin overexpression, but inhibited by suprabasin knock-down. Moreover, we demonstrated that upregulation of suprabasin activated the Wnt/β-catenin signaling pathway and led to nuclear localization of β-catenin and upregulation of Cyclin D1 and c-Myc. Together, our results suggest that suprabasin plays an important oncogenic role in promoting proliferation and tumorigenesis of ESCC.

Esophageal cancer is the eighth most common cancer and the sixth most frequent cause of cancer-related death in the world^1^,^2^,^3^. Esophageal squamous cell carcinoma (ESCC) is the main subtype of esophageal cancer, comprising approximately 70% of esophageal cancer cases, although occurrence rates vary widely with geographic location^1^,^4^,^5^,^6^. According to a report from the American Cancer Society, the prognosis of esophageal cancer is relatively poor, with survival rates of 40% in patients with early-stage (I and II) disease; survival rate decreases dramatically in patients showing advanced clinical symptoms to 21% in patients with T4 tumors and cancers that have spread to proximal lymph nodes, and 4% in patients in which cancer has spread to organs or lymph nodes further away from the tumor including all M1 (stage IV) cancers. Due to a lack of effective diagnostic methods for ESCC, most patients are diagnosed at the advanced stage, and most unfortunately die within the first year of diagnosis^7^,^8^,^9^,^10^. Therefore, identifying more effective diagnostic and prognostic markers is of great urgency.

The suprabasin gene, originally identified as a gene expressed in mouse and human differentiating keratinocytes, is an epidermal differentiation marker and a potential cornified envelope precursor^11^,^12^. Park and colleagues detected suprabasin in the suprabasal layers of the epithelia of the tongue, stomach and epidermis, and its expression was induced in differentiating primary cultured human keratinocytes, indicating a potential role in epidermal differentiation [12]. Interestingly, suprabasin is highly expressed in highly invasive glioblastoma multiform cells, suggesting it may contribute to cancer progression^13^. Furthermore, suprabasin is also found to be upregulated in tumor endothelial cells (TEC) compared with normal endothelial cells, and silencing inhibited both TEC migration and tube formation^14^. Suprabasin is reported to play an important role in maintaining the anchorage-dependent and -independent cell proliferation in salivary gland adenoid cystic carcinoma (ACC)^15^, and is a novel oncogene candidate involved in promoting carcinogenesis in non-small cell lung carcinoma (NSCLC)^16^. Collectively, these studies suggest that suprabasin is an oncogene that contributes to the progression and development of various tumors. However, studies on the expression, clinical significance and biological function of suprabasin in ESCC have not been reported.

In the current study, we found that suprabasin was upregulated in ESCC and associated with clinicopathological characteristics of ESCC patients. Overexpression of suprabasin promoted the proliferation and tumorigenicity of ESCC cells, both *in vitro* and *in vivo*. Furthermore, we demonstrated that upregulation of suprabasin enhanced Wnt/β-catenin signaling activity, and the stimulatory effects of suprabasin on proliferation and tumorigenesis of ESCC cells were drastically reduced by Wnt/β-catenin pathway inhibition. These results suggest that suprabasin plays an important role in promoting proliferation and tumorigenesis of ESCC and represents a novel prognostic marker for this devastating disease.

## Results

### Suprabasin is upregulated in ESCC

Analysis of high-throughput data from the Cancer Genome Atlas (TCGA; http://cancergenome.nih.gov/) database (Normal, n = 9; Tumor, n = 70) determined that suprabasin was significantly upregulated in ESCC tissues compared with normal tissues (*P* = 0.0033; Fig. 1a). Consistently, both suprabasin mRNA and protein levels were upregulated in 11 tested ESCC cell lines compared with normal human esophageal epithelial cells, and in all eight ESCC samples compared with paired adjacent noncancerous tissues (ANT) (Figs 1a–c and 2a,b). Additionally, suprabasin upregulation was further confirmed by IHC assays of the 8 paired ESCC and noncancerous tissue samples (Supplementary Fig. 1a,b). These results suggest that suprabasin is overexpressed in ESCC.

### Suprabasin is correlated with clinicopathological characteristics of ESCC patients

To explore the relationship between suprabasin expression and ESCC progression, 8 normal esophageal tissues and 170 paraffin-embedded archived clinical ESCC specimens (stage I, 10 cases; stage IIa, 74 cases; stage IIb, 15 cases; stage III, 62 cases; stage IV, 9 cases) were examined by IHC assay (Supplementary Table 1). Suprabasin expression was detected in almost all tumor specimens and expression was high in all stages of ESCC compared with normal esophageal tissues (Fig. 2c,d; Supplementary Tables 1–2). The correlation between suprabasin expression and the clinicopathological characteristics of ESCC was explored and showed a positive correlation between suprabasin expression and tumor clinical stage (*P* < 0.001), T classification (*P* < 0.001), N classification (*P* < 0.001), M classification (*P* = 0.016), and pathological differentiation (*P* < 0.001) (Fig. 2c,d and Supplementary Table 2). Spearman analysis further confirmed the correlation between suprabasin expression and clinical stage (r = 0.575, *P* < 0.001), T classification (r = 0.325, *P* < 0.001), N classification (r = 0.532, *P* < 0.001), histological differentiation (r = 0.512, *P* < 0.001), and tumor size (r = 0.183, *P* = 0.017; Supplementary Table 3). Taken together, these results strongly indicate that increased suprabasin expression is correlated to ESCC progression.

Statistical analysis also revealed a correlation between suprabasin expression and patient vital status (r = 0.412, *P* < 0.001; Supplementary Tables 2 and 3) and survival time (r = -0.619, *P* < 0.001; Supplementary Table 3). Log-rank testing and Kaplan–Meier analysis showed that higher suprabasin expression led to shorter survival, while lower suprabasin expression resulted in longer survival (*P* < 0.001; Fig. 2e). Moreover, we found that patients with higher suprabasin expression survived for a significantly shorter time than those with low expression in stages I and II (n = 84, *P* < 0.001) stages III and IV (n = 86, *P* = 0.001; Supplementary Fig. 2a), and in T1–T2 (n = 52, *P* < 0.001) and T3–T4 (n = 118, *P* < 0.001; Supplementary Fig. 2b). Importantly, higher expression of suprabasin led to shorter survival in both subgroups (lymph node–positive: n = 93, *P* < 0.001; lymph node–negative: n = 77, *P* < 0.001; Supplementary Fig. 2c). Univariable and multivariable Cox regression analysis showed that suprabasin expression might serve as an independent predictor of ESCC prognosis (*P* < 0.001; Supplementary Table 4).

In addition, we further analyzed the correlation between the clinicopathological characteristics of ESCC and suprabasin expression based on the computer-generated MOD. As shown in the Supplementary Table 5, suprabasin expression was significantly correlated with tumor clinical stage (*P* <  0.001), T classification (*P* < 0.001), N classification (*P* < 0.001). Furthermore, log-rank testing and Kaplan–Meier analysis showed that higher suprabasin expression led to shorter survival, while lower suprabasin expression resulted in longer survival (*P* < 0.001; Supplementary Fig. 2a). Moreover, univariable and multivariable Cox regression analysis showed that suprabasin expression might serve as an independent predictor of ESCC prognosis (*P* = 0.030; Supplementary Table 6). These results further supported the link between of suprabasin upregulation and progression and poor prognosis in ESCC.

### Suprabasin promotes cell proliferation of ESCC *in vitro*

As suprabasin expression was correlated with ESCC progression, we investigated possible effects of suprabasin on the tumorigenic activity of ESCC cells. KYSE510 and KYSE180 cells in which suprabasin was overexpressed or silenced, respectively, were established (Fig. 3a, Supplementary Fig. 3a). MTT assay showed that suprabasin overexpression increased the growth rate of ESCC cells, while silencing had the opposite effect (Fig. 3b, Supplementary Fig. 3b). Meanwhile, overexpressing suprabasin in ESCC cells resulted in a greater number of colonies that were larger in size, while colonies formed by suprabasin-silenced cell were fewer in number and smaller, compared to controls (Fig. 3c, Supplementary Fig. 3c). Furthermore, we found that BrdUrd-positive cells was significantly elevated in suprabasin-transduced ESCC cells but decreased in suprabasin-silenced cells (Fig. 3d, Supplementary Fig. 3d). Meanwhile, we found that overexpressing suprabasin dramatically promoted the cell growth and proliferation of NEEC1, further supported the oncogenic role of suprabasin (Supplementary Fig. 4a–c). These results suggest that suprabasin promotes the proliferation of ESCC cells *in vitro*.

### Suprabasin upregulation enhances the tumorigenicity of ESCC cells *in vitro* and *in vivo*

To examine the effect of suprabasin on ESCC cell tumorigenicity, an anchorage-independent growth assay was performed and showed that suprabasin-transduced ESCC cells formed a larger number and larger colonies than control cells, while suprabasin inhibition had the opposite effect (Fig. 4a, Supplementary Fig. 3e). The oncogenic role of suprabasin in ESCC progression was further examined using an *in vivo* tumor model. As shown in Fig. 4b–d, tumors formed from suprabasin-overexpressing ESCC cells were larger and heavier than vector-control tumors. In contrast, suprabasin-silenced tumors were smaller and weighed less than control cells (Fig. 4b–d, Supplementary Fig. 3f–h). Collectively, these results further support the notion that suprabasin contributes to ESCC tumorigenicity both *in vitro* and *in vivo*.

### Overexpressing suprabasin activates Wnt/β-catenin signaling

To investigate the underlying mechanism of suprabasin-associated promotion of ESCC progression, gene set enrichment analysis (GSEA) of the published esophageal cancer dataset (TCGA) was performed. As shown in Fig. 5a, suprabasin expression was significantly correlated with Wnt/β-catenin pathway, which suggests that suprabasin might be involved in activation of Wnt/β-catenin signaling. Indeed, overexpressing suprabasin significantly increased TCF/LEF activities in ESCC cells, while silencing had the opposite effect (Fig. 5b). Consistently, subcellular fractionation revealed a significant nuclear accumulation of β-catenin in suprabasin-overexpressing ESCC cell lines, whereas suprabasin-silenced cells contained less β-catenin in the nucleus (Fig. 5c). In addition, target genes downstream of the Wnt/β-catenin signaling pathway including *AXIN2*, *CTLA4*, *CCND1*, *FGFs*, *FRA1*, *ITF2*, *MMP7*, *JUN*, *LEF1*, *MYC* and *TCF1* were dramatically upregulated in cells overexpressing suprabasin and downregulated in silenced cells (Fig. 5d). Consistently, western blotting analysis revealed that protein expression of Cyclin D1 and c-Myc was significantly increased in suprabasin-overexpressing cells but decreased in suprabasin-silenced cells (Fig. 5e). However, overexpression of suprabasin dramatically reduced, but downregulation of suprabasin increased, expression of phosphorylated β-catenin (phospho S33 ± S37). Moreover, we found that overexpression of suprabasin dramatically decreased, but downregulation of suprabasin increased, the expression of phosphorylated β-catenin (Fig. 5e). Importantly, the stimulatory effects of suprabasin on proliferation and tumorigenesis of ESCC cells were drastically reduced upon treatment with a Wnt/β-catenin pathway inhibitor, both *in vitro* and *in vivo* (Fig. 5f–h), suggesting that functional Wnt/β-catenin activation is vital to the biological effects of suprabasin in ESCC cells. The expression of GSK3β and phosphorylated GSK3β were further examined. The results showed that suprabasin increased the phosphorylation of GSK3β, while downregulation of suprabasin decreased expression of phosphorylated GSK3β (Supplementary Fig. 5a). Meanwhile, we found that GSK-3β inhibitor BIO-A treatment significantly disrupted the inhibited effect of suprabasin downregulation on Wnt/β-catenin pathway activity in ESCC cells, cell proliferation and anchorage-independent growth capacity (Supplementary Fig 5b–d), demonstrating that the oncogenic effect of suprabasin on Wnt/β-catenin activity in ESCC cells might be through inhibition of GSK-3β.

## Discussion

The present study reports, for the first time, the association between suprabasin expression and ESCC progression. We found that suprabasin was upregulated in ESCC and its expression is correlated with multiple ESCC malignant symptoms. Specifically, higher suprabasin expression was associated with advanced disease progression, shorter survival, and poor prognosis. Moreover, overexpression of suprabasin dramatically promoted the proliferation and tumorigenicity of ESCC cells via activation of Wnt/β-catenin signaling. Therefore, our results demonstrated an oncogenic role of suprabasin in ESCC progression and pathogenesis.

ESCC is the most prevalent subtype of esophageal cancer, and is characterized by poor prognosis and high mortality rate. It is more common in developing countries, especially China, where both ESCC morbidity and mortality are the highest in the world^17^,^18^,^19^. Since the high mortality stems from the lack of effective methods for detecting the disease in the early stages, there is an urgent need to explore reliable methods for diagnosing ESCC^7^. To this end, multiple genes have been reported as ESCC diagnostic markers. For example, Slug has been reported as a diagnostic biomarker and predictor of poor prognosis, and disease recurrence is likely if Slug is upregulated^20^. The histone demethylase gene amplified in squamous cell carcinoma 1 (GASC1) is upregulated in ESCC and is a potential prognostic and predictive marker^21^. Herein, we showed that suprabasin was overexpressed in ESCC and expression was correlated with a number of ESCC clinical features. Suprabasin may therefore prove to be a valuable diagnostic and prognostic biomarker of ESCC, which might be helpful for early detection and hence improving survival.

The Wnt/β-catenin signaling pathway plays an essential role in diverse physiological processes, including various malignancies^22^,^23^,^24^. In conjunction with its role in tumor formation and progression, the Wnt/β-catenin signaling pathway presents an attractive cancer diagnostic and therapeutic target. The present study demonstrated that Wnt/β-catenin signaling is activated by suprabasin, suggesting this pathway may mediate the biological effects in ESCC. Expression of target genes downstream of the β-catenin signaling pathway, such as *AXIN2*, *CTLA4*, *CCND1*, *FGFs*, *FRA1*, *ITF2*, *MMP7*, *JUN*, *LEF1*, *MYC* and *TCF1*, was upregulated by suprabasin, further confirming the link to Wnt/β-catenin signaling. This signaling pathway has been reported to play a role in various cancer-related processes including cell growth, invasion and metastasis, apoptosis, differentiation and stem cell development^23^,^25^,^26^,^27^. It may therefore be of interest to explore other biological activities of suprabasin that may be related to malignant features of ESCC. Our study also found that the tumors formed by suprabasin-overexpressing ESCC cells exhibited increased percentages of microvascular density (MVD) whereas the tumors formed by suprabasin–silenced tumors displayed decreased MVD, indicating a potential function of suprabasin on ESCC angiogenesis (Supplementary Fig. 6).

Previously, suprabasin was found to be epidermal-specific expression, specific to the suprabasal-differentiated layers of inter-follicular trunk and tail epidermis and was detected in the stratified layers in the tongue and palate. In situ hybridization of different human tissues showed suprabasin expression in the esophagus, uterus, and thymus^11^. Recently, it was reported suprabasin was upregulated in TEC compared with NEC (normal endothelial cells). Moreover, Chad and colleagues found suprabasin was upregulated in NSCLC^16^. Meanwhile, it has been reported that suprabasin has a potential transmembrane domain in the amino-terminal region and a series of glycine and histidine rich short tandem repeats in the central domain^11^. N-terminal hydrophobic sequence in suprabasin has been discussed as a potential transmembrane domain and suprabasin is regarded as stratified epithelium-specific secreted protein^12^. The immunofluorescence and western blotting data of Moffatt’s study strongly supported the secretory nature of suprabasin^28^. Consistent with previous reports, our present study found that suprabasin was overexpressed in ESCC cells and tissues, compared with normal control, and suprabasin protein almost expressed in the suprabasal-layers as previous reported.

Suprabasin was first reported as a novel tumor endothelial cell marker, and the correlation between suprabasin and tumor progression has recently received greater attention. Suprabasin knock-down inhibited TEC migration and tube formation capability^14^. Shao and colleagues found that suprabasin is upregulated in salivary gland ACC, and is important for maintaining anchorage-dependent and -independent growth and the invasive and metastatic capability^15^. As a newly identified gene, little is known regarding the function of suprabasin regulation in tumor development, including in ESCC. In the present study, suprabasin expression was found to be correlated with tumor clinical stage, T and N classification, histological differentiation, and tumor size. We also found that overexpressing suprabasin leads to promotion of ESCC cell proliferation and tumorigenesis, both *in vitro* and *in vivo*, indicating an important oncogenic function in ESCC development.

Although upregulation of suprabasin has been observed in various tumors, little is currently known about its regulatory mechanism. Analysis of the suprabasin promoter region using the CONSITE program predicted two typical NF-κB-responsive elements, suggesting that NF-κB might be contributes to Suprabasin upregulation. Indeed, it has been reported that Ca (2+) or 12-O-tetradecanoylphorbol-13-acetate treatment in cultured primary mouse epidermal keratinocytes resulted in the induction of suprabasin^11^. Furthermore, shao *et al.* found that suprabasin is hypomethylated in salivary adenoid cystic carcinoma and suprabasin transcription is significantly upregulated induced by 5-aza-2′-deoxycytidine^15^. Gene amplification is a typical mechanism through which solid tumors activate oncogenes, and we noticed that suprabasin was localized at chromosomal region 19q13, which was shown to be amplified in pancreatic, ovarian, breast, cervical, gastric and lung cancers^29^,^30^,^31^,^32^,^33^,^34^. Moreover, amplification of the 19q13 chromosomal locus was found to be associated with clinicopathological parameters and patient survival^29^. Therefore, it may be of great interest to explore the regulatory mechanism of suprabasin upregulation in ESCC, and work towards this end has already commenced in our laboratory.

## Methods

### Cell lines and cell treatment

The ESCC cell lines, including KYSE30, KYSE140, KYSE180, KYSE410, KYSE510, KYSE 520, ECa109, 108Ca, TE-1, EC18 and HKESC1 were grown in DMEM medium (Invitrogen, Carlsbad, CA, USA) supplemented with 10% fetal bovine serum (Invitrogen) and 100 μg/ml penicillin, and 100 μg/ml streptomycin (Invitrogen) at 37 °C in a humidified atmosphere containing 5% CO_2_. Cell treatment: Wnt/β-catenin response inhibitor IWR-1-endo (10 μM; sc-295215, Santa Cruz, Dallas, Texas, USA) and GSK-3β inhibitor BIO-A (1 μM, Selleck, Boston, MA, USA) were dissolved in dimethyl sulfoxide (DMSO).

### Patient information and tissue specimens

This study was conducted on eight pairs of matched ESCC tissues and the non-cancerous adjacent tissues to the malignant lesion and a total of 170 paraffin embedded samples, which were histopathologically and clinically diagnosed with ESCC from 2001–2006 at the Sun Yat-sen University Cancer Centre, underwent esophageal cancer resection (Supplementary Table 1). Eight ESCC biopsy samples and their adjacent matching noncancerous (ANT) esophageal tissues were frozen in liquid nitrogen and stored. The eight fresh normal esophageal tissues were taken from the adjacent noncancerous esophageal tissue, which is over 5 cm from the cancerous tissue and was examined by routine histopathological analysis. The information of these eight ESCC and normal esophageal tissue samples are collected form Clinical stage II: 3 and stage III: 5. All samples were obtained from the Tissue Bank of Sun Yat-sen University Cancer Centre and coded anonymously in accordance with local ethical guidelines. We obtained approval from the Review Board of Sun Yat-sen University Cancer Centre and informed consent in accordance with the Declaration of Helsinki. ESCC specimens were staged in accordance with American Joint Cancer Committee/Union Internationale Contre le Cancer (UICC/AJCC) classification guidelines. The grading and histopathology subtyping of ESCC specimens were based on WHO criteria.

### RNA extraction, reverse transcription and quantitive RT-PCR (qRT-PCR)

Total RNA from cells and fresh surgically obtained tumor tissues and their adjacent noncancerous tissues was extracted using the Trizol reagent (Invitrogen) according to the manufacturer’s instruction. The extracted RNA was pretreated with RNase-free DNase, and 2 μg of RNA from each sample was used for cDNA synthesis primed with random hexamers. The qRT-PCR primers to amplify *suprabasin* were designed using Primer 5. *suprabasin* primers were as follows: forward, 5′-TCTGCTCTGCGTCCTGATAG-3′; reverse, 5′-GAAATGAAAGGCACCCAAA A-3′; *Glyceraldehyde 3-phosphate dehydrogenase* (*GAPDH*) primers included: forward, 5′-ATTCCACCCATGGCAAATTC-3′; reverse, 5′-ATTCCACCCATGG CAAATTC-3′. qRT-PCR was carried out using the FastStart Universal SYBR Green Master (Roche, Toronto, ON, Canada) on the Bio-Rad CFX96 qRT-PCR detection system (Bio-Rad Laboratories, Hercules, CA, USA). Expression data were normalized to the geometric mean of housekeeping gene GAPDH to control the variability in expression levels and calculated as 2^−[(Ct of *suprabasin*) – (Ct of *GAPDH*)]^, where Ct represents the threshold cycle for each transcript.

### Plasmids and retroviral infection

A SBSN1 expression construct was generated by subcloning PCR-amplified full-length human SBSN1 cDNA into the pMSCV vector. For depletion of SBSN1 to silence endogenous SBSN1, short hairpin RNA (shRNA) oligonucleotides were cloned into the pSuper-retro-puro vector to generate pSuper-retro- SBSN1-RNAi. Stable cell lines expressing SBSN1 and SBSN1-shRNA were generated via retroviral infection using HEK293T cells as previously described^35^ and selected with puromycin (0.5 μg/ml) 48 h after infection, for 10 days.

### Western blotting analysis

Western blotting was performed according to a previously reported method^36^. Total protein was extracted from whole cells and 20 μg of isolated protein was separated by SDS-PAGE and electroblotted onto a PVDF membrane (Bio-Rad Laboratories). The membrane was probed with monoclonal mouse anti-suprabasin antibody (Sigma, Saint Louis, MO, USA), and anti-β-catenin, anti-phospho-β-catenin (phospho S33 ± S37), anti-c-myc, anti-CyclinD1, anti-p84 antibodies (Abcam, Cambridge, MA, USA), anti-GSK3β and anti-phospho-GSK3β antibodies (Cell Signaling, Danvers, MA, USA). The membranes were then stripped and re-probed with an anti-GAPDH antibody (Cell Signaling) as a loading control.

### Immunohistochemistry (IHC) assay

Paraffin-embedded tissues were analyzed using immunohistochemical staining according to previously described methods^36^,^37^, with suprabasin antibody (Sigma) with a dilution rate of 1:100. The degree of immunostaining of formalin-fixed, paraffin-embedded sections was reviewed and scored separately by two independent pathologists uninformed of the histopathological features and patient data of the samples. Scores were determined by combining the proportion of positively stained tumor cells and the intensity of staining. Scores, given by the two independent pathologists who blinded for the experimental data, were combined into a mean score for further comparative evaluation. Tumor cell proportions were scored as follows: 0 (no positive tumor cells); 1 (<10% positive tumor cells); 2 (10–35% positive tumor cells); 3 (35–75% positive tumor cells) and 4 (>75% positive tumor cells). Staining intensity was graded according to the following standard: 1 (no staining); 2 (weak staining = light yellow); 3 (moderate staining = yellow brown) and 4 (strong staining = brown). The staining index (SI) was calculated as the product of the staining intensity score and the proportion of positive tumor cells. Using this method of assessment, the expression of suprabasin in ESCC was evaluated by the staining index (scored as 0, 1, 2, 3, 4, 6, 8, 9 or 12). Staining index score > =6 was identified as high expression, while score <6 was low expression.

Results of IHC staining of tumor and normal tissues were quantitative analyzed with the AxioVision Rel.4.6 computerized image analysis system (Carl Zeiss, Oberkochen, Germany). The stained sections were evaluated at 200×  magnification, and 10 representative staining fields of each section were analyzed to obtain the mean optical density (MOD), which represents the strength of staining signals as measured per positive pixels, as previously reported^38^,^39^,^40^,^41^. In brief, stained slides were evaluated at ×200 magnification using the SAMBA 4000 computerized image analysis system with Immuno 4.0 quantitative program (Image Products International, Chantilly, VA, USA). Ten representative staining fields per tumor sample were analyzed to determine the MOD, which represents the concentration of the stain as measured per positive pixels in the whole tissue. A negative control in each staining batch was used for background subtraction in the quantitative analysis. The MOD data were statistically analyzed using the *t*-test to compare the average MOD difference between different groups of tissues; *P* < 0.05 was considered significant.

### 3-(4, 5-Dimethyl-2-thiazolyl)-2, 5-diphenyl-2H-tetrazolium bromide (MTT) assay

Cells (2 × 10^3^/well) were seeded in triplicate wells of 96-well plates. At each time point, cells were stained with 100 μl sterile MTT dye (0.5 mg/ml, Sigma) for 4 h at 37 °C, followed by removal of the culture medium and addition of 150 μl of DMSO (Sigma). The absorbance was measured at 570 nm, with 655 nm as the reference wavelength. All experiments were performed in triplicates.

### Colony formation assay

Cells (1 × 10^3^/well) were plated on a 6-well plate and cultured for 10 days. The colonies were fixed with 10% formaldehyde for 15 min and stained with 1.0% crystal violet for 5 min. All experiments were performed in triplicate.

### Bromodeoxyuridine labeling and immunofluorescence (BrdUrd incorporation assay)

Cells were plated on coverslips (Thermo Fisher Scientific, Waltham, MA, USA ) and allowed to settle for 24 hours, incubated with bromodeoxyuridine (BrdUrd) for 1 h and stained with anti-BrdUrd antibody (Sigma) according to the manufacturer’s instruction. Gray level images were acquired under a laser scanning microscope (Nikon Co., Tokyo, Japan).

### Anchorage-independent growth assay

DMEM medium containing 10% FBS and 0.33% agar was plated in 6-well plates and allowed for the agar to solidify. The cells were trypsinized and 2 × 10^3^ cells per well were mixed with medium containing 10% FBS and 0.66% agar, followed with plating on the prepared 6-well plates. After 10–14 days incubation at 37 °C in a humidified atmosphere containing 5% CO_2_, colony sizes were measured using an ocular micrometer. The colonies >0.1 mm in diameter were scored. All experiments were performed in triplicate.

### Xenografted tumor model

All experimental procedures were approved by the Institutional Animal Care and Use Committee of Sun Yat-sen University. BALB/c-nu mice (4–5 weeks of age), purchased from the Center of Experimental Animal of Guangzhou University of Chinese Medicine, were randomly divided into two groups (n = 5/group). One group of mice was inoculated subcutaneously with KYSE510/Vector cells (5 × 10^6^) in the left dorsal flank and with KYSE510/suprabasin cells (5 × 10^6^) in the right dorsal flank per mouse. Another group was inoculated subcutaneously per mouse with KYSE510/RNAi-Vector cells (5 × 10^6^) in the left dorsal flank and with KYSE510/suprabasin-RNAi cells (5 × 10^6^) in the right dorsal flank. Tumors were examined twice weekly; length, width, and thickness measurements were obtained with calipers and tumor volumes were calculated. Tumor volume was calculated using the equation (L × W^2^)/2. On day 30, tumors were detected by an IVIS imagining system (Caliper), then animals were euthanized, tumors were excised and weighed.

### Luciferase reporter assay

Cells (5 × 10^4^) were seeded in triplicate wells of 24-well plates and allowed to settle for 12 hours. 100 ng of reporter plasmids containing wild-type (CCTTTGATC; TOPflash) or mutated (CCTTTGGCC; FOPflash) T cell factor (TCF)/LEF DNA binding sites (Upstate Biotechnology, Lake Placid, NY, USA) plus 10 ng pRL-TK Renilla luciferase normalization control (Promega) were cotransfected using Lipofectamine 2000 (Invitrogen). Luciferase and Renilla signals were measured 48 hours after transfection by using the Dual Luciferase Reporter Assay Kit (Promega, Madison, WI, USA) according to manufacturer’s instruction. All experiments were performed in triplicate.

### Statistical analysis

Pearson’s Chi-square test and Spearman correlation analysis were also applied in studying the relationship between suprabasin expression and patient age, gender, tumor stage, TNM classification, histological differentiation, tumor size, and vital status. Survival curves for both suprabasin-high and -low patients were plotted using the Kaplan–Meier method, and statistical differences were compared using a log-rank test. Univariate and multivariable survival analysis was performed using Cox regression analysis. A *P*-value of less than 0.05 was considered statistically significant. All statistical analyses were performed using the SPSS statistical software package.

## Additional Information

**How to cite this article**: Zhu, J. *et al.* Overexpression of Suprabasin is Associated with Proliferation and Tumorigenicity of Esophageal Squamous Cell Carcinoma. *Sci. Rep.* **6**, 21549; doi: 10.1038/srep21549 (2016).

## Supplementary Material

Supplementary Information

## Figures and Tables

**Figure 1:** Increased suprabasin expression in ESCC cells. (**a**) Suprabasin is upregulated in ESCC (*P* = 0.0033; TCGA database). (**b**) The mRNA expression of suprabasin is upregulated in ESCC cell lines, analyzed by real-time PCR analysis. *GAPDH* served as the control. Bars represent the mean ± SD of three independent experiments. *P < 0.05. (**c**) The expression of suprabasin protein is upregulated in ESCC cell lines, compared to NEECs (normal human esophageal epithelial cells), analyzed by Western blotting analysis. GAPDH served as the loading control.

**Figure 2:** Suprabasin expression increases in ESCC tissues and correlates with ESCC progression. (**a,b**) Suprabasin expression increased in ESCC tissues (T), compared to the paired adjacent non-tumor tissue (ANT) specimens from eight patients, determined by real-time PCR analysis (**a**) and western blotting analysis (**b**). (**c**) Representative images of IHC analysis of ESCC specimens (clinical stage I–IV tumors) compared with normal esophageal tissue (Upper, 200×; Lower, 400×). (**d**) Statistical analysis of the mean optical density (MOD) of suprabasin staining in normal esophageal tissue and ESCC specimens at different clinical stages. (**e**) Kaplan–Meier curves of univariate analysis (log-rank) of overall survival for all patients with low versus high suprabasin expression. Bars represent the mean ± SD of three independent experiments. *P < 0.05.

**Figure 3:** Suprabasin promotes cell proliferation of ESCC *in vitro*. (**a**) Western blotting analysis of suprabasin expression in ESCC cell lines stably expressing or silencing suprabasin. (**b**) Suprabasin promotes growth rate of ESCC cells, determined by MTT assay. (**c**) Representative micrographs (left) and quantification (right) of colonies formed by the indicated cells as determined by colony formation assays. (**d**) Representative micrographs (left) and quantification (right) of the BrdUrd incorporation assay in the indicated cells. All experiments were performed with KYSE510 and KYSE180 cells stably overexpressing or silencing suprabasin. Bars represent the mean ± SD of three independent experiments. *P < 0.05.

**Figure 4:** Upregulation of suprabasin enhances the tumorigenicity of ESCC cells *in vitro* and *in vivo*. (**a**) Representative micrographs (left) and quantification (right) of colonies formed by the indicated cells, determined by anchorage-independent growth ability assays. (**b**) Representative images of the tumors from all mice in each group. (**c**) Tumor volumes were measured on the indicated days. (**d**) Mean tumor weights of all mice in each group. All experiments were performed with KYSE510 and KYSE180 cells stably overexpressing or silencing suprabasin. Bars represent the mean ± SD of three independent experiments. *P < 0.05.

**Figure 5:** Overexpressing suprabasin activates the Wnt/β-catenin signaling pathway. (**a**) GSEA analysis showing the correlation between suprabasin expression and Wnt/β-catenin signaling in the published breast cancer dataset (TCGA database). (**b**) Suprabasin activates the Wnt/β-catenin signaling activity, measured by luciferase assay of TCF/LEF transcriptional activity in the indicated cells. (**c**) Nuclear expression of β-catenin in indicated ESCC cell lines, determined by Western blotting using p84 as a nuclear marker. (**d**) Real-time PCR analysis of Wnt/β-catenin signaling pathway downstream genes expression, including *AXIN2*, *CTLA4*, *CCND1*, *FGFs*, *FRA1*, *ITF2*, *MMP7*, *JUN*, *LEF1*, *MYC* and *TCF1* mRNAs in the indicated ESCC cells. (**e**) Western blotting of phosphorylated β-catenin (phospho S33 ± S37), β-catenin, Cyclin D1 and c-Myc in ESCC cells. GAPDH was used as the loading control. (**f**,**g**) Quantification of colonies determined by colony formation (**f**) and anchorage-independent growth assays (**g**), after cells treated with IWR-1-endo (Wnt/β-catenin response inhibitor, 10μM) or vehicle control. (**h**) Representative images of the tumors from all mice in each group. Bars represent the mean ± SD of three independent experiments. *P < 0.05.
